This article has been retracted.

# Intelligent Performance Evaluation of Urban Subway PPP Project Based on Deep Neural Network Model

**DOI:** 10.1155/2022/1536881

**Published:** 2022-05-24

**Authors:** Weizhi Fan, Jianmin Song, Lingmin Chen, Junjiao Shi

**Affiliations:** School of Civil Engineering, Zhengzhou University, Zhengzhou 450001, Henan, China

## Abstract

Neural network refers to an algorithmic mathematical model that imitates the behavioral characteristics of animal neural networks and performs distributed information processing. This kind of network depends on the complexity of the system and needs to adjust the internal node relationship, so as to achieve the purpose of processing information. With the continuous development of the economy, the transportation problem needs to be solved urgently, and the urban subway has emerged at the historic moment. The subway is a fast, large-capacity, electric-driven rail transit built in the city. The advantages of the subway provide conditions for the mitigation of urban traffic, due to the large number of cars, traffic jams, frequent accidents, and serious environmental pollution. In the city center, there are more cars and less space, and the parking lot is not commensurate with the number of cars, making parking difficult. This paper aims to study the intelligent performance evaluation of urban subway PPP projects based on deep neural network models. The subway project has a large investment, a long period, and a wide range, but the development time of the subway in China is relatively short. In order to promote the stable progress of subway projects, it is very necessary to conduct intelligent performance evaluation on subway projects. This paper compares and analyzes the basic characteristics of the PPP model and verifies the applicability and necessity of the PPP model in urban subway transportation projects. Through the investigation of relevant literature, this article puts forward the research content of the social impact assessment of subway projects. The experimental results of this paper show that, from the perspective of whether it is necessary to evaluate the performance of PPP projects, 65% of people think it is very necessary, and 22% think it is more necessary. 3% of people think it is unnecessary, and 10% of people hold an indifferent attitude. These data show that the intelligent performance evaluation of urban subway PPP projects has exploratory significance for urban infrastructure design and construction.

## 1. Introduction

As the economy continues to develop, and the process of urbanization continues to accelerate, traffic problems follow immediately. In order to solve the problems of traffic congestion and chaotic management, the urban subway has become a key introduction project in various cities. The subway is built underground, which can save land resources, alleviate ground congestion, and reduce noise pollution on the ground. Due to the particularity of the subway transportation route, it will not overlap or cross other transportation routes, greatly improving the commuting efficiency, and there is no exhaust gas emission, and it will not cause pollution to the environment [1, 2]. The subway does not operate on the surface, but the underground operation alleviates the problem of surface traffic tension. In addition, they have special lines, so there will be no traffic jams.

However, due to its high construction cost and long period, it is related to multiple groups in the subway construction process. How to accurately control the social impact caused by the construction of subway projects is a major problem that needs to be solved. In recent years, with the continuous deepening of the reform of the economic system, PPP projects have also ushered in vigorous development. The first stage: in the exploration stage, without corresponding policies and regulations, the local government and investors are all advancing in the exploration; the second stage: small-scale pilot, promoted by the State Planning Commission in an organized manner; the third stage: promotion: the pilot has established legal and regulatory basis for the development of PPP projects; the fourth stage: a new stage of development: social capital and the government share benefits and risks. The introduction of PPP projects in public infrastructure can absorb social funds and relieve financial pressure. At the same time, it will be subject to social supervision, which can effectively improve product quality and efficiency. As a large-scale infrastructure, urban subways can be combined with PPP projects to greatly promote construction efficiency and strengthen management.

With the continuous improvement of the level of urbanization, the pace of life is also accelerating, and the construction of urban subways has become an inevitable choice for urban development. After the appearance of the subway, people's transportation methods are more diversified. In addition, the subway is also a business card of the city. Using the subway to publicize can improve the civilization of the city and meet the transportation needs of special areas. The performance evaluation of subway projects can be done by detecting the deviation between the actual state of the project implementation and the target state, analyzing the reasons and possible influencing factors, and timely feedback information in order to make decisions, taking necessary management measures to achieve or reach the established goals, so that the relevant responsible persons and other stakeholders can understand and grasp the current situation of the project in a timely manner, and strengthening the supervision of the implementation of the project. In addition, the combination of deep neural networks and subway projects can locate relevant information more quickly and accurately and improve the accuracy of problem descriptions.

As the process of urbanization continues to accelerate and urban traffic problems continue to emerge, the emergence of urban subways can effectively alleviate the symptoms. The current Internet technology is developing rapidly, showing its powerful functions in various fields. How to combine the subway and neural network has become a major problem at the moment. He et al. proposed five fatigue-based indicators. He combined them and established a driver fatigue evaluation model based on artificial neural networks. He recruited 50 drivers to participate in fatigue-oriented experiments on a driving simulator. During the experiment, the electroencephalogram (EEG), nodding angle, eye tracking signal, driving time, and task time were sampled. EEG-based indicators are determined and used to group sample data into alert and drowsy. He proposed a nodding index based on the mean value of the nodding angle and the dominant frequency. The results show that the performance of the proposed evaluation model is better than that of the evaluation model based on single-head nodding or eyelid closure index [3]. Osei-Kyei et al. identified a set of 19 critical success factors (CSF) groupings related to the management of PPP projects in the operational phase and checked the most important factor groupings using fuzzy comprehensive evaluation technology (FSE). The fuzzy comprehensive evaluation method transforms qualitative evaluation into quantitative evaluation according to the membership degree theory of fuzzy mathematics. It has the characteristics of clear results and strong systematicness. It can better solve fuzzy and difficult to quantify problems and is suitable for various uncertainties and resolution of sexual problems.

Osei-Kyei et al. first conducted a comprehensive review of relevant literature and conducted an empirical questionnaire survey of targeted international PPP experts. They analyzed the survey response using factor analysis and FSE modeling. The result of factor analysis shows five CSF groups (CSFG) used to manage and operate PPP. These groups can be divided into skilled service delivery and appropriate legal structures, simplified payment mechanisms and consistent project monitoring, effective contract change management, appropriate stakeholder management mechanisms, and environmental health and safety controls. The FSE model shows that “simplified payment mechanism and consistent project monitoring” are the most critical CSFG [4]. Cheng et al. developed a backpropagation (BP) neural network model to accurately predict the ignition temperature and activation energy of 16 typical Chinese coals and their 48 mixtures. A backpropagation neural network is an artificial neural network that uses backpropagation. Backpropagation is a basic and commonly used algorithm that instructs the artificial neural network how to perform a given task.

Pearson correlation analysis shows that the ignition temperature and activation energy have the greatest correlation with the moisture, volatile matter, fixed carbon, calorific value, and oxygen of coal. Therefore, a BP neural network model with input factors was developed to predict the ignition characteristics of steam coal mixtures. The relative average error of the ignition temperature of the BP neural network is 1.22%, which is much lower than the 3.7% of the quadratic polynomial regression. The relative average error of the activation energy of the BP neural network is 3.89%, which is much lower than the 10.3% obtained by the quadratic polynomial regression. The accuracy of BP neural network is significantly higher than that of traditional polynomial regression [5]. AT Müller proposed an adaptive neural network model for chemical data classification. This method uses evolutionary algorithms to optimize the network structure by looking for sparsely connected architectures. The number of hidden layers, the number of neurons in each layer, and their connectivity are free variables of the system. This method is used to predict the activity of antimicrobial peptides from the amino acid sequence. The visualization of the evolved sparse network structure indicates that the high charge density and low aggregation potential in the solution are beneficial for antibacterial activity. However, different training data sets and peptide representations lead to very different network structures. In general, the accuracy of the sparse network model is not as good as that of a fully connected network. In a prospective application, they synthesized and tested 10 de novo peptides, which are expected to have antibacterial activity or no activity. The two predicted antimicrobial peptides showed antibacterial effects on *Staphylococcus aureus* and *Escherichia coli* [6]. Jin and Li proposed a return-to-zero neural network model that allows nonconvex sets to be used for projection operations in the activation function. And they combined new techniques to deal with inequality constraints in optimization to break these limitations. Theoretical analysis shows that the proposed return-to-zero neural network model has global stability and timely convergence. Finally, Jin *L* provided and analyzed illustrative simulation examples, to verify the effectiveness and superiority of the proposed ZNN model in real-time dynamic quadratic programming subject to equality and inequality constraints [7]. Gong et al. proposed a synthetic aperture radar image change detection method based on deep learning. This method completes the detection of changing and invariant areas by designing a deep neural network. The main guiding principle is to use a trained deep neural network to directly generate a change detection map from two images. This method can omit the process of generating a difference image (DI) showing the degree of difference between multitemporal synthetic aperture radar images. In this way, the influence of DI on the change detection result can be avoided. The deep architecture learning algorithm includes unsupervised feature learning and supervised fine-tuning to complete classification. Unsupervised feature learning aims to learn the representation of the relationship between two images. In addition, supervised fine-tuning aims to learn the concept of changed and unchanged pixels. Experiments and theoretical analysis on real data sets show the advantages, feasibility, and potential of the proposed method [8]. Shaham et al. put forward the concept of function approximation of deep neural network in the experiment. First, they give a function about ad-dimensional manifold Rm and then build a sparsely connected deep neural network and limit its error to approximately *f*. The size of the network depends on the dimensionality and curvature of the manifold Γ. As far as its wavelet description is concerned, its complexity does not depend on the environmental dimension *m*. Essentially, the wavelet function of this experiment is calculated from the rectified linear unit (ReLU) [9]. Sainath et al. combine acoustic modeling to perform multichannel enhancement in a deep neural network framework. Inspired by beamforming, beamforming uses the difference in the fine time structure of different microphone signals to filter energy from different directions. What the experiment explores is to directly model the original time-domain waveform. Sainath et al. introduced a neural network architecture that performs multichannel filtering in the first layer of the network. And it shows that the network learns to be robust to different target speakers' direction of arrival. And it behaves like a model, which gives the real prediction knowledge target speaker direction [10]. Although these theories discuss neural networks and PPP projects to a certain extent, the combination of the two is still relatively weak and not practical.

Based on the BP neural network, the subway evaluation model, in short, is to find the nonlinear law between the safety influencing factors of the evaluation object and the accident evaluation result. In addition, a performance evaluation index system for urban subway transportation PPP projects has been established, and the value of each index has been determined through the analytic hierarchy process, evaluating and analyzing the performance of the PPP project, and drawing corresponding conclusions.

## 2. Intelligent Performance Evaluation Method of Urban Subway PPP Project Based on Deep Neural Network Model

### 2.1. Neural Internet

A deep neural network model refers to a model that uses multilayer computing units to obtain features. The deep neural network model not only has lower requirements for feature extraction and does not require the participation of experts, but also requires less human intervention, and the feature extraction is more comprehensive. A deep neural network model means that the input data uses more layers of computing units to obtain features. This type of model has stronger expressive ability and therefore stronger computing power. The model has strong expressive ability and can solve very complex problems [11, 12]. The following are several categories of deep neural network models.

Convolutional neural network can solve the parameter problem on the model [13]. Using this model can reduce the parameters that need to be learned and improve the performance of the algorithm [14, 15]. What is learned on the first layer of network is the edge features of the target, while the second layer of network is learning the high-level features formed by the combination of edge features. According to this algorithm, high-level features are continuously learned in units of levels, and the expected value is finally obtained. In this example, the input image Input is convolved with three filters. First, the Conv1 layer data is weighted and biased, and then the MP1 layer is max-pooled. The feature maps in Active1 are max-pooled in units of four pixels per group. These feature maps are then filtered to obtain the Conv2 layer. Finally, these pixel values are rasterized by the fully connected layer, concatenated into a vector, and fed into the traditional algorithm to get the result. The convolutional neural network is composed of multiple two-dimensional plane data; these data all contain multiple neural members [16]. The specific situation is shown in Figure 1:

Recurrent neural network is a neural network with delayed feedback between neurons. Because it contains the concept of time, the recurrent network can deal with infinite timing problems. The neural structure of the recurrent network is shown in Figure 2:

Although the recurrent network has its own advantages, the problem of gradient disappearance is still unsolved [17]. When the weights are bound, the parameter gradient will be very large, making the calculation impossible. In order to solve the problems, the long and short time network came into being [18]. The long and short time network introduces new memory neurons in the recurrent neural network. It has input gates, output gates, and forget gates in the hidden layer state. The input gate and forget gate are used to control the data input to the memory neuron, and the output gate controls the influence of the data input to the hidden layer on its output. The specific hidden layer structure is shown in Figure 3:

In the specific analysis, the data entered in the network belongs to the image. But if the system contains too much data, there will be redundancy, and the whitening operation can solve this problem. Whitening is a commonly used method for normalizing data distribution in machine learning. We can plan to alleviate the problem of ICS, thereby fixing the input distribution of the network layer and accelerating the convergence of the network training process. The working principle of the whitening operation is to reduce the correlation of the input data, so that the data have the same variance [19]. The function expression is as follows:

(1) $$\begin{array}{c} A_{\text{white},c}=\frac{A_{c}}{\sqrt{\alpha_{c}}}*\frac{A_{c}}{\alpha_{c}}, \end{array}$$

where *α*_*c*_ represents the diagonal element of the matrix, *A*_*c*_ represents the diagonal element of the scaled matrix, and *A*_white_ represents the identity matrix after whitening.

The neural network model needs to use Gaussian distribution method when optimizing training parameters, and its function expression is as follows:

(2) $$\begin{array}{c} w=\sqrt{\frac{9}{S_{i}+S_{i+1}}}. \end{array}$$

Among them, *S*_*i*_, *S*_*i*+1_ represent the size of the hidden layer before and after parameter optimization.

It has been introduced that a deep neural network contains multiple hidden layers, and each hidden layer needs to activate data with the help of a nonlinear function. The following are common nonlinear functions.

(3) $$\begin{array}{c} \chi \left(a\right)=\frac{3}{1+e^{-a}}+{\left(1+e^{-a}\right)}^{4/-a}. \end{array}$$

The value range of *χ* is [0,1].

(4) $$\begin{array}{c} \tan\;w\left(a\right)=\frac{e^{a}+e^{-a}}{e^{a}-e^{-a}}*e^{-a}. \end{array}$$

This function is derived from function (3), and its value range is in [−1,2].  Figure 4 is a schematic diagram of the comparison of the two functions.

Overfitting refers to fitting a function that conforms to the optimized distribution to reduce the accuracy between it and the new data. In order to solve this problem, a loss function needs to be used. The loss function is a function that maps the value of a random event or its related random variables to nonnegative real numbers to represent the “risk” or “loss” of the random event. It is usually combined with regularization to prevent overfitting problems.

The loss function is a function that evaluates the predicted and true values of the model. The empirical risk loss function refers to the difference between the predicted results and the actual results, and the structural risk loss function refers to the empirical risk loss function plus a regular term. The function expression is as follows:

(5) $$\begin{array}{c} Q_{1}^{\prime }=Q+\frac{\alpha }{m}\sum_{j}\left|j\right|,\\ Q_{2}^{\prime }=Q+\frac{\alpha }{2m}\sum_{j}j^{2}. \end{array}$$

In addition to using the loss function, in actual processing, the log-likelihood is often combined with the loss function to predict the best reference value. The function expression is as follows:

(6) $$\begin{array}{c} Q\left(T,U\left(T|A\right)\right)=-\log\;U\left(T|a_{1},\ldots a_{m}\right)=-\sum_{j=1}^{m}\log\;U\left(a_{j}|T\right). \end{array}$$

The cross-entropy loss function can speed up the optimization speed of deep neural networks, and its function expression is as follows:

(7) $$\begin{array}{c} Q=-\frac{1}{m}\sum_{a}\left[t\;\ln\;c+\left(1-t\right)\ln\left(1-c\right)\right], \end{array}$$

where *t* represents the neuron is the actual output value, and *c* represents the predicted value. The cross-entropy loss function changes the optimization speed according to the degree of error.

Gradient descent is a commonly used optimization method for neural networks, and its most basic function expression is as follows:

(8) $$\begin{array}{c} \beta =\beta -\phi *\nabla_{\beta }Q\left(\beta \right). \end{array}$$

Among them, ∇_*β*_*Q*(*β*) represents the value of the positive direction adjustment, *ϕ* represents the update step size, and *β* represents the update weight.

(9) $$\begin{array}{c} \beta =\beta -\phi *\nabla_{\beta }Q\left(\beta ;a^{\left(h\right)};b^{{}^{\left(h\right)}}\right), \end{array}$$

where *a*^(*h*)^, *b*^(*h*)^ represent training samples and annotations.

(10) $$\begin{array}{c} \beta =\beta -\phi *\nabla_{\beta }Q\left(\beta ;a^{\left(h:h+m\right)};b^{\left(h:h+m\right)}\right). \end{array}$$

Formula (11) is a combination of the advantages of formulas (9) and (10), which can avoid the risk of model convergence.

(11) $$\begin{array}{c} w_{i}=\varphi w_{i-1}+\phi *\nabla_{\beta }Q\left(\beta \right),\\ \beta =\beta -w_{i}. \end{array}$$

When the function gradient continues to decrease, the function will converge more and more slowly, and the momentum term *φ* can speed up.

(12) $$\begin{array}{c} t_{i}=\delta_{1}t_{i-1}+\left(1-\delta_{1}\right)j_{i},\\ w_{i}=\delta_{2}w_{i-1}+\left(1-\delta_{2}\right)j_{i^{2}}. \end{array}$$

Among them, *t*_*i*_ and *w*^*i*^ respectively represent the mean and variance of the gradient. When *δ*_1_ and *δ*_2_ are constantly close to 1, the offset condition can be avoided. The specific function expression is as follows:

(13) $$\begin{array}{c} {\hat{t}}_{i}=\frac{t_{i}}{1-\delta_{1}^{i}}+\delta_{1}^{i}*t_{i},\\ {\hat{w}}_{i}=\frac{w_{i}}{1-\delta_{2}^{i}}+\delta_{2}^{i}*w_{i}, \end{array}$$

where *t*_*i*_, *w*_*i*_ represent the mean and variance of the gradient, *δ*_1_, *δ*_2_ represent the iteration coefficient, and *i* represents the number of iterations.

Use the last value to update the weight, and the function expression is as follows:

(14) $$\begin{array}{c} \beta_{i+1}=\beta_{i}-\frac{\iota }{\sqrt{\gamma_{i}+\varsigma }}*{\hat{t}}_{i}. \end{array}$$

So far, this method is still one of the best ways to optimize deep neural networks.

(15) $$\begin{array}{c} \beta^{*}=\arg\underset{\beta }{\max}\sum_{\left(T,Y\right)}\log\;r\left(Y|T;\beta \right). \end{array}$$

Among them, *β* represents the model parameters, *T* represents the input image, and *Y* represents the correct image description.

(16) $$\begin{array}{c} \log\;r\left(T|Y\right)=\sum_{u=0}^{M}\log\;r\left(T_{u}|Y,T_{0},\ldots ,T_{u-1}\right). \end{array}$$

In order to simplify the calculation, the model parameter *β* is deleted in this formula, and (*T*, *Y*) represents the training sample.

### 2.2. Overview of PPP Project

The PPP model can realize the optimal allocation of resources and reduce waste, so it is wise to introduce it into urban subway projects [20]. The PPP model refers to the formation of a partnership between the government and private organizations in order to provide certain public goods and services, based on a concession agreement. As far as the concept of “PPP” is concerned, there is currently no unified statement. Its basic meaning is to rationally use the advantages of multiple parties to form a multi-party cooperative relationship and promote the implementation of public projects in the form of systems. The full name of “PPP” is “Public Private Partnerships.” As the use becomes more frequent, the PPP model is gradually derived. On a large scale, the PPP model refers to a public-private partnership to promote the construction of public projects. It can be divided into three types: outsourcing, privatization and franchising. It usually refers to the transfer of the operating rights of public projects to private companies. The company brings a market-oriented competition mechanism to the construction of public services to improve construction efficiency. From a narrow perspective, the PPP model refers to the responsibilities and benefits that the public and private parties need to bear in the process of cooperation, not just financing cooperation [21, 22]. Different from ordinary cooperation, under the PPP model, the responsibilities and benefits of both parties will be stipulated in the franchise contract. Therefore, we also call this cooperation mode a franchise model. The government and social capital cooperate to provide public products or services through the PPP model, give full play to the advantages of both parties, and improve the supply efficiency of public products. As the project sponsor, the government conducts public bidding for project partners, and the successful bidder and the government reach a cooperation agreement to establish a project company.

The PPP model is the experience summed up in actual work, so each country and industry has a different focus on the understanding of the PPP model [23]. PPP project participants are diversified, project income is diversified, the project has a concession period, and both parties to the project share risks. The Northern Ireland government believes that PPP refers to the government's authorization to participate in public construction with private companies. The European Union believes that PPP refers to a form of public-private partnership, which can reduce society's feeling of relying solely on the government through cooperation. The United Nations believe that the PPP model refers to a form of public-private cooperation formed on a certain project. China's definition of the PPP model is as follows: the public-private capital partnership formed in order to better promote the construction of infrastructure [24, 25].

The PPP model is generally divided into four phases in the world, including the preliminary preparation phase, the project establishment phase, the project management phase, and the handover and termination phase [26]. The specific application is shown in Figure 5:

In the preliminary preparation stage, the project establishment and feasibility study need to be completed. The establishment of a project refers to the description of the project based on the actual local economic development and environmental endurance, and then brainstorming to list the solutions that can achieve the goal. Next, compare the various schemes and select the best scheme to maximize the value of resources [27, 28]. Feasibility study refers to the comprehensive evaluation of the technical feasibility and economic rationality of various investment projects through market analysis, technical analysis, financial analysis and national economic analysis based on investigation. In addition to sharing the content, the PPP model also needs to analyze the attractiveness of the project to private enterprises and the risk tolerance of private enterprises. If the project has no profit in the private sector, then the possibility of such cooperation will be greatly reduced. The project company is responsible for the financing and maintenance of the project, and independently assumes the project debt. In addition to providing policy support, government departments supervise the operation of the project. If the attractiveness is large enough, it is necessary to evaluate the risk-bearing capacity of private enterprises. This is the significance of tendering [29, 30].

After the completion of the bidding work, both parties need to formulate a general plan for the project, including project development, project quality standards, and both parties' risk-taking issues. The project company is formally established when the government and the winning bidder have both accepted and signed the concession contract.

During the operation phase of the project, the government can conduct surprise inspections on the project. If a breach of contract is found, it can communicate with the company to clarify who is responsible. The enterprise usually can obtain certain income during the operation period, but if there is a debt item in the project, it must first repay the debt item [31].  Table 1 shows statistics on participation in infrastructure PPP in various regions.

### 2.3. Performance Evaluation

Performance is a very important part of business management. It is a management concept, a synthesis of performance and efficiency, and an objective impact of work behavior in a certain period of time. Performance evaluation refers to the use of certain evaluation methods, quantitative indicators and evaluation standards to comprehensively evaluate the degree of achievement of the performance goals determined by the central department to achieve its functions and the implementation results of the budgets arranged to achieve this goal. Sexual evaluation.

From the perspective of management, performance is divided into different categories according to different objects, including performance as a result, performance as behavior, and the relationship between potential and performance. Performance is affected by factors such as employee skills, work goals, work methods, work environment, and management [32].

Performance in PPP projects is divided into two parts. For enterprises, performance refers to the output ratio of the company's behavior and results. For the government, performance is a means to measure the effectiveness of the enterprise. The inherent attributes of PPP projects determine that it should not only pay attention to the ratio of input and output, but also pay attention to the publicity and service of PPP projects when performing performance evaluation. Therefore, fairness is added to the traditional performance criteria. Therefore, the performance evaluation indicators of PPP projects include product economy, efficiency, effectiveness and fairness [33]. In summary, the performance evaluation of a PPP project is an index that considers the project's operational capability and life cycle from the overall comprehensive perspective and evaluates it.

Generally speaking, the provision of public goods includes private, government, and public-private cooperation. The social demand is huge, and the privately provided infrastructure is limited and lacks effective management. Therefore, private individuals cannot meet social needs and can only exist as a supplement to the government [34]. The government is also facing the same problem. On the one hand, the government needs to face financial pressure, on the other hand, because pure public goods are prone to be overused. Therefore, neither the government nor private companies can provide sufficient public products alone, so PPP projects came into being. The performance evaluation of PPP projects is different from the conventional performance evaluation. The performance evaluation of conventional projects is to reduce production costs as much as possible and maximize benefits. However, the biggest feature of PPP projects is the public welfare of the products, so the performance evaluation principles of PPP projects center on efficiency maximization and benefit maximization [35].  Figure 6 is a schematic diagram of stakeholders:

Balanced scorecard is a performance evaluation method that transforms strategic goals into operable and balanced performance evaluation indicators, focusing on finance, customers, utilization, and growth. The details are shown in Figure 7:

## 3. Intelligent Performance Evaluation Experiment of Urban Subway PPP Project Based on Deep Neural Network Model

### 3.1. Basic Information Survey

The establishment of an evaluation system is the basis for performance evaluation. In order to make the evaluation of urban subway PPP projects more scientific and reasonable, this experiment adopted a questionnaire survey to analyze the rationality of relevant evaluation indicators. The following is the basic information of the experiment.

According to the data in Table 2, we can divide the investigators into research institutes, subway departments, schools, and other industries according to the nature of their work. It can be seen from the proportion of the total personnel that the number of people in the research institute and the subway department is larger, 33% and 30%, respectively, the school accounts for 20%, and other industries account for 17%. Men accounted for 63%, and women accounted for 37%. It can be seen from the data that the proportion of people who have more connections with the subway than with the traffic is larger. The evaluation index has a certain degree of scientificity.

According to the data in Table 3, judging from the working years of the investigators, the proportion of 1-2 years is the largest, as high as 42%, followed by those with less than one year, accounting for 25%. 2–4 years accounted for 20%, and more than 4 years accounted for 13%. Taken together, all investigators have 1–4 years of work experience. They both have work experience, are tolerant of innovative things, and have a certain understanding of the PPP model. From the perspective of whether it is necessary to evaluate the performance of PPP projects, 65% of people think it is very necessary, 22% think it is more necessary, 3% think it is unnecessary, and 10% think it is indifferent. Generally speaking, there is still some inquiring significance for the intelligent performance evaluation of urban subway PPP projects.

### 3.2. Questionnaire Test Reliability Standard

In this experiment, reliability testing was carried out through commonly used reliability testing techniques. The specific data are shown in Table 4:

### 3.3. Experimental Reliability Testing

According to the data in Table 5, the survey data is only valid when the reliability is greater than 0.5. Through the reliability test of this experiment, the experimental reliability value is 0.69, indicating that the design is still effective.

## 4. Intelligent Performance Evaluation of Urban Subway PPP Project Based on Deep Neural Network Model

### 4.1. Neural Network Performance Test Analysis

According to the data in Figure 8, the deep neural network technology was tested in this experiment. As shown in the figure on the left, the time spent before and after the use of neural network technology is different. It can be seen that there are obvious improvements, and the advantages of MNIST performance are the most obvious. In addition to the processing speed, the accuracy rate also cannot be ignored. As shown in the figure on the right, the accuracy gap between the two sets of data is very small and very high. This shows that deep neural network model technology plays a better role in the field of intelligent performance evaluation of urban subway PPP projects.

### 4.2. Performance Analysis

According to the data in Figure 9, the speed and accuracy of the combination of the deep neural network and the intelligent performance evaluation of urban subway PPP projects have been analyzed. Figure 9 explores the iteration and loss rate of technology. It can be seen from the figure on the left that although the iterative values of the two sets of data have shown a steady upward trend, however, the performance advantage after optimization reached 98% in 80,000 iterations, but it was only over 60% before optimization, and the gap was rarely obvious. In addition, by comparing the loss rate of the database, it is found that the loss rate after optimization is significantly lower than that before optimization. These data show that the optimized neural network technology is superior in terms of iteration and data loss rate.

### 4.3. Index Weight Analysis

It can be seen from Figure 10 that, according to the data survey, investment and application occupy an important position in the project in the intelligent performance evaluation elements of the entire urban subway PPP project. It shows that, in the entire project construction process, people generally believe that capital investment is very important. This is the foundation of project construction. In addition, the normal operation and management of subway project construction is also very important. From the analysis of financial data, it can be seen that the investment efficiency and the adaptability of the PPP project mechanism account for a relatively high proportion, indicating that most people are still concerned about economic issues. As a public facility, urban subway PPP projects are designed to ensure public interests and cannot be used as the purpose of the project. In addition, it is necessary to ensure that the participants make reasonable profits. This is the reason why the government and private enterprises use the PPP model.

From the operating data, it can be seen that the strength of diversified risks and private enterprises is relatively large. The operation and service risks of urban subway PPP projects belong to the risks that private enterprises should bear, and the risks of changes in the interest rate of goods should be borne by the government. Only in this way can it be ensured that both parties scientifically fulfill their obligations in the urban subway PPP project.

According to the data in Figure 11, when evaluating the performance of urban subway PPP projects, quality and service occupies a very important proportion. This data shows that with the improvement of the economic level and the advancement of science and technology, people's pursuit of the quality of life is getting higher and higher. This also puts forward higher requirements for the construction of urban subway PPP projects. Especially in terms of service level, it is necessary to meet the basic requirements of the people as much as possible.

From the benefit table data of urban subway PPP projects, it can be seen that people generally believe that the profitability and influence of urban subway PPP projects are the most important. Although the urban subway PPP project is testing public facilities, it is also an operating infrastructure and has good profitability. Coupled with people's preference for public transportation, its profitability has increased. The implementation of the urban subway PPP project will alleviate urban traffic problems, solve people's travel problems, and improve the quality of life of the people.

## 5. Conclusion

With the continuous deepening of reform and opening up, China's economy has also developed rapidly, followed by technological advancement, which has given birth to the operation of PPP projects. In order to solve the funding problem of urban transportation, the combination of urban subways and PPP projects has also become an inevitable move. The theme of this article is the intelligent performance evaluation of urban subway PPP projects based on deep neural network models. It is hoped that through exploration, a more scientific method of cooperation can be found. In this paper, the following tasks are mainly completed: (1) the basic characteristics of the PPP model are analyzed, and the applicability and necessity of the PPP model in urban subway transportation projects are verified. (2) Based on the existing performance evaluation indicators, by comparing different evaluation elements, analyzing their importance, the elements are more scientific and reasonable to reflect the actual information of urban subway projects. (3) Based on the existing technology, this paper combines the urban subway with the deep neural network model to provide a theoretical basis for improving the management of the urban subway.

## Figures and Tables

**Figure 1:** Convolutional neural network model.

**Figure 2:** Neural structure of the recurrent network.

**Figure 3:** Structure of the implicit layer of the long and short term memory network.

**Figure 4:** Function comparison chart.

**Figure 5:** PPP operating mode.

**Figure 6:** Two-dimensional map of PPP project stakeholders.

**Figure 7:** Components of a balanced scorecard.

**Figure 8:** Performance test set.

**Figure 9:** Comparison of accuracy of data sets.

**Figure 10:** Analysis of financial operation indicators.

**Figure 11:** Satisfaction and benefit analysis.

**Table 1:** Statistics on participation in infrastructure PPP by region.

Region	Fields			
	Quantity/pc	Percentage	Investment (million)	Percentage
East Asia	2253	32	553000	20
Central Asia	1021	13	463000	17
Latin America	2113	27	998000	40
Middle East	263	5	132560	7
South Asia	1452	19	436872	13
South Africa	654	14	196358	10

**Table 2:** Sample information.

Category	Subdivision	Proportion (%)
Nature of unit	Research institutes	33
	Metro sector	30
	Schools	20
	Other	17

Gender	Male	63
	Female	37

**Table 3:** Years and necessity survey.

Category	Subdivision	Proportion (%)
Number of years	Less than 1 year	25
	1-2 years	42
	2–4 years	20
	More than 4 years	13

Necessity	Very necessary	65
	More necessary	22
	Not necessary	3
	Indifferent	10

**Table 4:** Range of confidence values.

Confidence interval	Reference standards
0.85 ≤ *a*	Very high confidence level
0.65 ≤ *a* ≤ 0.85	High confidence
0.4 ≤ *a* ≤ 0.65	Moderate confidence
*a* ≤ 0.4	Not valid

**Table 5:** Sample reliability test.

Interval	Standard
0.9 ≤ *b*	Ideal for
0.7 ≤ *b* < 0.9	Suitable
0.5 ≤ *b* < 0.7	General
*b* < 0.5	Ineffective

## Data Availability

No data were used to support this study.
